RETRACTED

# SqueezeNet for the forecasting of the energy demand using a combined version of the sewing training-based optimization algorithm

**DOI:** 10.1016/j.heliyon.2023.e16827

**Published:** 2023-06-03

**Authors:** Noradin Ghadimi, Elnazossadat Yasoubi, Ehsan Akbari, Mohammad Hosein Sabzalian, Hamzah Ali Alkhazaleh, Mojtaba Ghadamyari

**Affiliations:** a Young Researchers and Elite Club, Ardabil Branch, Islamic Azad University, Ardabil, Iran; b College of Technical Engineering, The Islamic University, Najaf, Iraq; c Department of Electrical Engineering, West Tehran Branch, Islamic Azad University, Tehran, Iran; d Department of Electrical Engineering, Mazandaran University of Science and Technology, Babol, Iran; e Smart Grid Laboratory (LabREI), Department of Systems and Energy, School of Electrical and Computer Engineering (FEEC), University of Campinas (UNICAMP), Campinas, Brazil; f College of Engineering and IT, University of Dubai, Academic City, 14143, Dubai, United Arab Emirates; g Department of Electrical Engineering, Shahid Beheshti University, 48512 Tehran, Tehran, Iran

**Keywords:** Energy demand forecasting, SqueezeNet, Combined sewing training-based optimization

## Abstract

With the introduction of various loads and dispersed production units to the system in recent years, the significance of precise forecasting for short, long, and medium loads have already been recognized. It is important to analyze the power system’s performance in real-time and the appropriate response to changes in the electric load to make the best use of energy systems. Electric load forecasting for a long period in the time domain enables energy producers to increase grid stability, reduce equipment failures and production unit outages, and guarantee the dependability of electricity output. In this study, SqueezeNet is first used to obtain the required power demand forecast at the user end. The structure of the SqueezeNet is then enhanced using a customized version of the Sewing Training-Based Optimizer. A comparison between the results of the suggested method and those of some other published techniques is then implemented after the method has been applied to a typical case study with three different types of demands-short, long, and medium-term. A time window has been set up to collect the objective and input data from the customer at intervals of 20 min, allowing for highly effective neural network training. The results showed that the proposed method with 0.48, 0.49, and 0.53 MSE for Forecasting the short-term, medium-term, and long-term electricity provided the best results with the highest accuracy. The outcomes show that employing the suggested technique is a viable option for energy consumption forecasting.

RETRACTED

## 1 Introduction

### 1.1 Problem statement

Energy as a resource of human activities is of vital importance in human life, and on this basis, all the countries of the world are seeking access to reliable and planned sources of energy. On the other hand, due to the non-renewability of fossil fuel sources, especially oil and gas sources, it has been several decades that the issue of replacing these types of energy and saving and optimal consumption of energy has been seriously considered in the economy of advanced countries, and very effective measures have been taken to optimize energy consumption [1]. As a result of preventing the rapid depletion of non-renewable energy sources, various research organizations and institutions, both governmental and private, have been implemented for this purpose in various countries, especially industrial countries, since the 1972s, to conduct research in the field of planning. Energy consumption and saving and optimizing it have been established and energy has been raised as one of the important and strategic issues in the economy of the nations of the world [2].

With the establishment of the electricity market in the power grid, electricity companies on the one hand, and distribution companies, which are considered energy buyers, on the other hand, need to be able to predict and present the hour-by-hour consumption of the entire network covered by them in the coming days. In addition, power plant production and operation management companies may also need load forecasting to forecast and offer prices [3]. In a developing country, with accurate forecasting, while improving the operation of the network under the cover of allocation of relevant crimes in the electricity market, it is possible to reduce the frequency of grid shutdown and prevention [4]. This load prediction is common in developed countries for periods shorter than a few minutes. In general, electricity networks have a wide range of types and types of consumers, which can be divided into household, industrial, commercial, general, and agricultural loads [5]. Load forecasting enables distribution companies to create a proper balance between production and demand to estimate the accurate price of electricity and manage the planning of production capacity [6]. The structure of load forecasting in distribution networks is divided into two parts: daily load forecasting and annual or mid-term load forecasting [7].

Short-term and medium-term load forecasting is generally done for periodic planning and is not very complicated [8]. But long-term forecasting is more difficult due to the long period of load forecasting and requires the use of complex mathematical and statistical methods. In various studies, the topic of load forecasting has been investigated in different periods.

RETRACTED

The literature shows that short-term load forecasting has attracted more attention than medium-term load forecasting [9]. Of course, the structure of algorithms and available information has also been more relevant in this regard. Forecasting has wide applications in power system control, unit sharing, economic load spreading, and the electricity market [10]. On the other hand, mid-term and short-term load forecasting, due to its vital features for planning and budgeting, have not been studied enough [11].

Recently, there has been a significant shift away from purely theoretical research and toward applied research to tackle issues that have no solution or cannot be handled easily [12]. Given this, there is a growing interest in the creation of model-free intelligent dynamic systems based on experimental data. Artificial Neural Networks (ANNs) are among the dynamic systems that can analyze empirical values [13]. They discover the law in the data.

In the last decade, different analytical or numerical techniques have been proposed in the field of forecasting science, in such a way that instead of presenting a mathematical model, these methods try to use a free model obtained from a series of experimental and practical data [14]. These techniques are often (in a way) modeled on human behavior, especially the behavior of the human brain, so they are known as artificial intelligence methods [15]. Among the major characteristics and advantages of these methods, we can mention their accuracy, resistance, flexibility, and ease of finding. Artificial intelligence components include neural networks [16], expert systems [17], metaheuristic algorithms [18], and fuzzy logic [19].

### 1.2 Background

With the increasing use of various loads and dispersed production units in the power system, the importance of accurate load forecasting has been widely recognized. It is crucial to analyze the system’s performance in real-time and respond appropriately to changes in the electric load to maximize the energy system’s efficiency. Long-term electric load forecasting enables energy producers to increase grid stability, reduce equipment failures and production unit outages, and ensure the reliability of electricity output.

### 1.3 Literature survey

Several methods have been proposed for electric load forecasting, including statistical models, machine learning techniques, and deep learning algorithms. However, most of these methods have limitations in terms of accuracy, computational efficiency, and scalability. For example, Romera et al. [20] studied monthly electricity requirement forecasts using neural networks and the Fourier series. The monthly Spanish electrical requirement series, which was achieved by ignoring the trend in the consumption series, is the subject of this study’s investigation into its periodic behavior. The periodic behavior is predicted using a Fourier series, while the trend is anticipated using a neural network. This is a novel hybrid approach. With less than 2% MAPE, satisfactory findings have been achieved, which are better than those attained when only neural networks or ARIMA were utilized for the same objective. The research was limited by the fact that the conclusions may not be generalizable to other nations or regions with different consumption patterns or environmental factors, that the forecasts' accuracy is greatly influenced by the caliber of the input data, and that there may be mistakes or data gaps that could impair the validity of the results. The hybrid technique utilized in the study may be computationally demanding, restricting its practical implementation in some contexts with limited resources. The assumptions proposed in the study may not reflect the intricate connections between trends and periodic behavior, resulting in inaccurate projections. Furthermore, the study only took into account monthly electricity needs, and it is unknown how the model would function at various periods (daily, weekly, etc.).

RETRACTED

Huang et al. [21] presented a new energy demand forecasting framework that used an optimal model with linear and quadratic forms. The model was optimized using an adaptive genetic algorithm and cointegration analysis based on historical annual data on electricity usage from 1985 to 2015. The model predicted that the annual growth rate of electricity demand in China will slow down, but due to population growth, economic growth, and urbanization, China will continue to demand about 13 trillion kilowatt hours in 2030. The model is more accurate and reliable than other single optimization methods.

Chen et al. [22] presented an improved energy demand forecasting model that uses the autoregressive distributed lag (ARDL) bounds testing approach and an adaptive genetic algorithm (AGA). The ARDL bounds analysis is used to select appropriate input variables, and the AGA is used to optimize coefficients of both linear and quadratic forms with various input variables. Historical annual data from 1985 to 2015 is used, and the simulation results show that the proposed model is more accurate and reliable than conventional optimization methods.

Ghanbari et al. [23] suggested an ant colony optimization-genetic algorithm approach for building knowledge-based expert approaches for energy demand forecasting. They created expert systems with the capacity to model and simulate fluctuations in energy demand under the influence of related factors using a novel methodology called “Cooperative Ant Colony Optimization Genetic Algorithm” (COR-ACO-GA). Utilizing three case studies of annual demand for electricity, natural gas, and petroleum products, they applied COR-ACO-GA to assess its functionality. The findings demonstrate that COR-ACO-GA offers results that are more accurate and consistent than those produced by artificial neural networks (ANN) and adaptive fuzzy neural inference systems (ANFIS). This information can assist decision-makers in formulating plans and making the right choices for the future. The limitations of the research were not explicitly stated, but possible limitations could include the generalizability of the findings, as the study only considered three case studies of annual demand for electricity, natural gas, and petroleum products, and the applicability of the methodology to other energy demand forecasting scenarios. Additionally, the study may have relied on assumptions and simplifications that may not accurately reflect the complex and dynamic nature of energy demand, and the computational requirements of the approach may be a limiting factor in practical implementation.

RETRACTED

Ahmad et al. [24] examined utility companies' use of machine learning-based models for forecasting short-term energy demand. They used machine learning-based models to predict the amount of energy needed by water source heat pumps in the future. Their findings showed that this analysis can help utilities prioritize energy-efficient improvements and facilities for investment by highlighting the impact of weather variables on building background electricity consumption and improving short- and medium-term power forecasting with scarce weather data. Do Energy predictions performed with the help of CDT, FitcKnn, LRM, and Stepwise-LRM models yielded results that were evaluated as 0044%, 0051%, 0776%, 0343%, and 7523%. 1 point 766, 12 points 317, and 5 points 969 respectively.

The limitations of the research were not explicitly stated, but possible limitations could include the generalizability of the findings to other energy demand forecasting scenarios, as the study focused specifically on predicting the energy demand of water source heat pumps. Additionally, the study may have relied on assumptions and simplifications that may not accurately reflect the complex and dynamic nature of energy demand, and it was unclear whether the machine learning-based models used in the study can be easily implemented in practical settings. The study also did not provide a detailed analysis of the limitations of the different machine learning models used, and it was unclear whether the findings can be replicated using different models or datasets.

RETRACTED

Su et al. [25] investigated a combined deep-RNN model and wavelet transform-based hourly natural gas requirement prediction approach. In this work, they proposed a reliable hybrid gas consumption approach. The wavelet transform was used to break the original series of gas loads into smaller and more manageable components to reduce the complexity of the prediction tasks. They used a multi-layer Bi-LSTM model LSTM model to create a deep learning method with RNN structure used to improve the structure of the deep learning model. The results of graphical analysis and analysis of numerical errors showed the superior efficiency of the presented model in forecasting hourly natural gas requirements.

The limitations of the research were not explicitly stated, but possible limitations could include the generalizability of the findings to other natural gas demand forecasting scenarios and the applicability of the proposed hybrid gas consumption approach to other types of energy forecasting. Additionally, the study may have relied on assumptions and simplifications that may not accurately reflect the complex and dynamic nature of energy demand, and it is unclear whether the deep-RNN model and wavelet transform-based approach used in the study can be easily implemented in practical settings. The study also did not provide a detailed analysis of the limitations of the different components of the proposed hybrid approach, and it was unclear whether the findings can be replicated using different models or datasets.

Ruiz et al. [26] investigated energy consumption forecasting. Our social lives depend heavily on buildings Using Elman neural networks and assessed optimization. To increase energy efficiency without compromising comfort or health, they proposed a method to forecast energy consumption in public buildings and thereby achieve energy savings. For intelligent systems to function and be planned, energy consumption forecasting is crucial. They suggest an elementary neural network forecast such consumption, and we employ a genetic algorithm to improve the weight of the models. The findings demonstrated that the suggested approach improved energy consumption forecast and enhanced the findings from earlier research.

The limitations of the research work were not explicitly stated, but possible limitations could include the generalizability of the findings to other types of buildings or energy forecasting scenarios, as the study focused specifically on public buildings. Additionally, the study may have relied on assumptions and simplifications that may not accurately reflect the complex and dynamic nature of energy demand in buildings, and it was unclear whether the Elman neural network-based approach used in the study can be easily implemented in practical settings. The study also did not provide a detailed analysis of the limitations of the genetic algorithm used to improve the weight of the models, and it is unclear whether the findings can be replicated using different models or datasets.

RETRACTED

In the literature, many approaches for predicting energy consumption were proposed. It is a randomness-based model for picking either the user data in the modeling or the NN training. When it comes to predicting energy use, researchers have routinely used artificial neural networks. When a neural network cannot execute on its own, optimization strategies such as metaheuristic algorithms must be utilized to improve training outcomes. When compared to a regular neural network, the optimized neural network model produces better results.

### 1.4 Challenges and motivation

Electric load forecasting poses several challenges, including uncertainty in load demand, variability in renewable energy generation, and the difficulty of modeling complex energy systems accurately. The motivation behind this study is to enhance the accuracy of long-term electric load forecasting by developing a new method that can overcome these challenges.

### 1.5 Contributions and novelties

The recommended approach involves modifying the weights throughout a neural network training session to get a faster convergence rate with excellent accuracy. Because of the aforementioned difficulties, we are motivated to use NN-based optimization for demand-side management in the smart network. Highly adaptable new electricity transmission networks must be constructed to satisfy current needs and enhance consumer profitability. To avoid abuse of the energy system by destroying electrical equipment, the model must estimate client demand. It must also be suitable for the design and construction of new power generation facilities. Therefore, the main contributions of this study can be highlighted by the following:

− The study uses SqueezeNet to forecast power demand at the user end.
− The structure of SqueezeNet is enhanced using a customized version of the Sewing Training-Based Optimizer.
− The proposed method is compared with other published techniques using a typical case study with short, long, and medium-term demands.
− Objective and input data are collected at intervals of 20 min.

### 1.6 Methodology

The study first uses SqueezeNet to obtain power demand forecasts at the user end. SqueezeNet is a deep learning architecture that has been previously used for image classification tasks. The structure of SqueezeNet is then enhanced using a customized version of the Sewing Training-Based Optimizer. This optimizer has been previously used in various deep-learning tasks and has shown improved performance compared to standard SGD.

RETRACTED

Next, the proposed method is compared with other published techniques using a typical case study with short, long, and medium-term demands. The previous research studies that are used for comparison are cited in the paper.

To collect objective and input data from customers, a time window is set up at intervals of 20 min, allowing for highly effective neural network training. The authors provide a detailed description of the data collection process in the paper.

Finally, the proposed method is evaluated and the results are presented, showing that it achieved the best results with the highest accuracy, with 0.48, 0.49, and 0.53 MSE for short-term, medium-term, and long-term electricity forecasting.

In conclusion, the authors have presented a detailed description of the methods used in the study and have cited relevant previous research studies where necessary, which would help readers replicate their results.

## 2 Combined sewing training-based optimization

### 2.1 Sewing training-based optimization (STBO)

The introduction and mathematical simulation of the optimization algorithm based on sewing training (STBO) are presented below:

#### 2.1.1 Main idea and inspiration of the STBO

The process of training novice tailors by the tailoring trainer is the central idea and source of motivation for the STBO Algorithm. First, a novice selects a sewing trainer to enhance her sewing abilities. Then sewing strategies are taught by the trainer. In the second stage, the trainer’s abilities are imitated by novice tailors and they attempt to increase their abilities to the level of their trainer. In the last stage, novice tailors increase their abilities by doing exercises. The process described as sewing training is an intelligent process that by mathematical simulation of this process, the suggested optimizer is inspired.

#### 2.1.2 Mathematical simulation of the STBO

Novice tailors and tailor trainers are individuals who constitute the population of the suggested STBO algorithm. The value of the decision variables is suggested through any individuals of the algorithm which indicates a candidate solution to the problem. Consequently, a vector and a matrix can express any individual and population of the STBO algorithm mathematically. The following equation represents the population of STBO as a matrix [27] Eqs. (1), (2), (3):

(1) $$Z={\left[\begin{array}{c} Z_{1}\\ \vdots \\ \begin{array}{c} Z_{i}\\ \vdots \\ Z_{N} \end{array} \end{array}\right]}_{N\times m}={\left[\begin{array}{ccc} \begin{array}{c} z_{1,1}\\ \vdots \\ \begin{array}{c} z_{i,1}\\ \vdots \\ z_{N,1} \end{array} \end{array} & \begin{array}{c} \cdots \\ \ddots \\ \begin{array}{c} \cdots \\ \ddots \\ \cdots \end{array} \end{array} & \begin{array}{ccc} \begin{array}{c} z_{1,j}\\ \vdots \\ \begin{array}{c} z_{i,j}\\ \vdots \\ z_{N,j} \end{array} \end{array} & \begin{array}{c} \ldots \\ \ddots \\ \begin{array}{c} \cdots \\ \ddots \\ \cdots \end{array} \end{array} & \begin{array}{c} z_{1,m}\\ \vdots \\ \begin{array}{c} z_{i,m}\\ \vdots \\ z_{N,m} \end{array} \end{array} \end{array} \end{array}\right]}_{N\times m}$$

where Z indicates the population matrix of the STBO, $Z_{i}$ indicates the $i^{th}$ STBO’s individual, N and m denote the number of STBO individuals and problem variables, the following equation defines the random initialization of the population individuals at the start of the algorithm [27]:

(2) $$z_{i,j}={lb}_{j}+r.\left({ub}_{j}-{lb}_{j}\right),i=1,2,\ldots ,N.\;j=1,2,\ldots ,m\text{.}$$

where $z_{i,j}$ denotes the value of the $j^{th}$ the variable specified by the $i^{th}$ STBO’s individual $Z_{i}$, r indicates a random amount between 0 and 1, ${ub}_{j}$ and ${lb}_{j}$ represent the upper and lower limits of the $j^{th}$ problem variable.

RETRACTED

Any STBO individual illustrates a candidate solution to the determined issue. Hence, the fitness function of the problem can be assessed based on the defined values through any candidate solution. The computed values for the fitness function are simulated based on the placement of candidate solutions in the problem parameters as follows:

(3) $$F={\left[\begin{array}{c} F_{1}\\ \vdots \\ \begin{array}{c} F_{i}\\ \vdots \\ F_{N} \end{array} \end{array}\right]}_{N\times 1}={\left[\begin{array}{c} F\left(Z_{1}\right)\\ \vdots \\ \begin{array}{c} F\left(Z_{i}\right)\\ \vdots \\ F\left(Z_{N}\right) \end{array} \end{array}\right]}_{N\times 1}$$

where F represents the fitness function vector and $F_{i}$ represents the fitness function value for the $i^{th}$ candidate solution. To analyze the obtained solutions and select the best solution from among the population, the fitness function values are evaluated. The finest individual in the population ($Z_{b}$) is the individual who has the finest value of the fitness function. In each iteration, the population of the algorithm is renewed and as a result, novel fitness function values are found. Therefore, the finest candidate solution is also renewed, which is more acceptable than all the former solutions. The approach of renewing solutions in STBO individuals are executed in three stages: (1) instruction, (2) emulation of the trainer’s abilities, and (3) assiduity in exercise.

RETRACTED

Stage 1: Instruction (exploration). The first stage of renewing STBO individuals is based on modeling the approach of choosing a sewing trainer and attaining sewing ability by novice tailors.

For any STBO individual as a novice tailor, whole different individuals with a more suitable value for the fitness function are assumed sewing trainers for that individual. The grouping of whole candidate individuals as the set of probable sewing trainers for any STBO individual $Z_{i}=1,2,\ldots ,N$, is specified as follows [27]:

(4) $${CSI}_{i}=\left\{Z_{k}|F_{k}<F_{I},k\varepsilon \left\{1,2,\ldots ,N\right\}\right\}\cup \left\{Z_{b}\right\}$$

where ${CSI}_{i}$ indicates the group of whole probable candidate sewing trainers for the $i^{th}$ STBO individual. When $Z_{i}=Z_{b}$ the probable candidate sewing trainer is $Z_{b}$ itself, that’s mean ${CSI}_{i}=\left\{Z_{b}\right\}$. After that, for any i∈[1,2,...,N], an individual from the group ${CSI}_{i}$ is chosen at random as the sewing trainer of the $i^{th}$ individual of STBO, and it is indicated as ${SI}_{i}$. The $i^{th}$ STBO individual learns sewing ability from this chosen trainer ${SI}_{i}$. As a result of the instruction of the population members by the trainers, the algorithm individuals can analyze various parts of the search space and identify the principal optimal part. The exploration capability in the global search of the suggested procedure is illustrated by the renewing stage of the STBO. At first, a novel location for any individual is created by the following equation and individuals of the population are renewed based on this stage of the algorithm.

(5) $$z_{i,j}^{p1}=z_{i,j}+r_{i,j}.\left({SI}_{i,j}-I_{i,j}.z_{i,j}\right)\text{,}$$

where $z_{i,j}^{p1}$ defines its $d^{th}$ dimension, $F_{i}^{p1}$ represents its fitness function value, $I_{i,j}$ indicates amounts that are chosen at random from the [1,2], and $r_{i,j}$ indicates a random amount between 0 and 1.

Eventually, if this novel location enhanced the fitness function value, it changes that individual’s former location. The following equation represents the condition of updating:

(6) $$Z_{i}=\left\{ \begin{array}{cc} Z_{i}^{p1}, & F_{i}^{p1}<F_{i};\\ Z_{i}, & else, \end{array}\right.$$

where the novel location of the $i^{th}$ STBO individual based on the first stage is indicated by $Z_{i}^{p1}$.

Stage 2: Emulation of the trainer’s abilities (exploration). The second stage of renewing STBO individuals is based on modeling novice tailors attempting to imitate the abilities of trainers. It is assumed that novice tailors want to increase their ability as much as possible and bring it to the level of a trainer. According to any optimization individual is a vector of the dimension m and any component illustrates a decision variable therefore, in this stage of the optimization, it is presumed that any decision variable indicates a sewing ability. Any member of STB optimization emulate $m_{s}$ abilities of the determined trainer, 1≤m_s≤m. This approach drives the individuals of the algorithm to various parts in the solution space, which illustrates the STBO exploration capability. The collection of variables that any optimization member emulates is defined in the following equation.

(7) $${SD}_{i}=\left\{d_{1},d_{2},\ldots ,d_{m}\right\}\text{,}$$

where ${SD}_{i}$ defines a m_s_− an assortment of the [1,2,...,m] , which indicates the collection of the indexes of decision variables (i.e., abilities) determined for emulation by the $i^{th}$ individual from the trainer and $ms=1+\frac{t}{2T}m$ is the numeral of abilities chosen to emulate, t indicates the iteration computer, and T is the numeral of iterations.

RETRACTED

The novel location for any STBO individual is computed based on the modeling of emulating these trainer abilities, utilizing the following formula [27]:

(8) $$z_{i,j}^{p2}=\left\{ \begin{array}{cc} {SI}_{i,j}, & j\varepsilon {SD}_{i}\\ z_{i,j}, & else \end{array}\right.$$

where $z_{i,j}^{p2}$ indicates the novel location created for the $i^{th}$ STBO individual based on the second stage in the $j^{th}$ dimension. This novel location substitutes the former location of the related individual if it enhances the value of the fitness function.

(9) $$Z_{i}=\left\{ \begin{array}{cc} Z_{i}^{p2}, & F_{i}^{p2}<F_{i}\\ Z_{i}, & else \end{array}\right.$$

where $Z_{i}^{p2}$ represents the fitness function value of $Z_{i}^{p2}$.

Stage 3: Assiduity in exercise (exploitation). The third stage of renewing STBO individuals is based on modeling novice tailoring exercises for enhancing sewing abilities. In this stage of the optimization process, a local search is executed near candidate individuals to discover the finest probable solutions around these candidate individuals. This stage of the STBO illustrates the exploitation sufficiency of the suggested algorithm in local search. For the mathematical expression of this step, a novel location near any individual of the STBO is created through the following equation.

(10) $$z_{i,j}^{p3}=\left\{ \begin{array}{cc} {lb}_{j}, & z_{i,j}^{*}<{lb}_{j}\\ z_{i,j}^{*}, & z_{i,j}^{*}\in \left[{lb}_{j},{ub}_{j}\right]\\ {ub}_{j}, & z_{i,j}^{*}>{ub}_{j} \end{array}\right.$$

where $z_{i,j}^{*}=z_{i,j}+({lb}_{j}+r_{i,j}\left({ub}_{j}-{lb}_{j}\right)/t$ and $r_{i,j}$ indicates a random amount between 0 and 1. Therefore, if the value of the fitness function enhances it substitutes the former location of the STBO individual as follows:

(11) $$Z_{i}=\left\{ \begin{array}{cc} Z_{i}^{p3}, & F_{i}^{p3}<F_{i};\\ Z_{i}, & else \end{array}\right.$$

where $Z_{i,j}^{p3}$ represents the novel-created location for the $i^{th}$ STBO individual based on the second stage of the optimization process, in the $j^{th}$ dimension, and $F_{i}^{p3}$ indicates its fitness function value.

RETRACTED

#### 2.1.3 Iteration approach and pseudo-code of STBO

By renewing all candidate solutions based on the first to third stages, the first iteration in the optimization process is performed. After that, the renewing approach is continued up to the final iteration of the algorithm, according to Eqs. (4), (5), (6), (7), (8), (9), (10), (11). Through the full execution of STB optimization, the finest candidate solution stored during the iteration of the algorithm is determined as the solution for the specified problem. The steps of the STB optimization execution are given as pseudo-code as follows:

**Table:** 

Algorithm 1. Pseudo-code of STBO
Start STBO. 1. Input the optimization problem information. 2. Set N and T. 3. Initialize the STBO individuals by (2) and generate vector F of the values of the fitness function by (3). 4. For t=1 to T. 5. For i=1 to N. 6. Stage 1: Training (exploration) 7. Specify the collection of candidate sewing trainers for the $i^{th}$ individual by (4). ${CSI}_{i}\leftarrow \left\{Z_{k}|F_{k}<F_{i},k\varepsilon \left\{1,2,\ldots .,N\right\}\right\}\cup \left\{Z_{b}\right\}$, 8. Select the sewing trainer ${SI}_{i}$ from ${CSI}_{i}$ for training sewing the $i^{th}$ STBO individual. 9. Compute the novel location for the $i^{th}$ STBO individual utilizing (5). $z_{i,j}^{p1}\leftarrow z_{i,j}+r_{i,j}.\left({SI}_{i,j}+I_{ij}.z_{i,j}\right)$. 8. Update the location of the $i^{th}$ STBO individual utilizing (6). 10. Stage 2: Imitation of the trainer’s abilities (exploration) 11. Compute ${SD}_{i}$ utilizing equation (7). 12. Compute the novel location of the $i^{th}$ STBO individual utilizing equation (8). $z_{i,j}^{p2}=\left\{ \begin{array}{cc} {SI}_{i,j}, & j\varepsilon {SD}_{i};\\ z_{i,j}, & else \end{array}\right.$. 13. Renew the location of the $i^{th}$ STBO individual utilizing (9). $Z_{i}=\left\{ \begin{array}{cc} Z_{i}^{p2}, & F_{i}^{p2}<F_{i};\\ Z_{i}, & else \end{array}\right.$. 14. Stage 3: Exercise (exploitation) 15. Compute the novel location for the $i^{th}$ STBO member utilizing (10). $z_{i,j}^{p3}=z_{i,j}+({lb}_{j}+r_{i,j}\left({ub}_{j}-{lb}_{j}\right)/t$. 16. Renew the location of the $i^{th}$ STBO individual utilizing (11). $Z_{i}=\left\{ \begin{array}{cc} Z_{i}^{p3}, & F_{i}^{p3}<F_{i};\\ Z_{i}, & else \end{array}\right.$. 17. End 18. Renew the finest candidate solution. 19. End 20. Output the finest candidate solution attained by STBO. End STBO.

RETRACTED

### 2.2 Combined sewing training-based optimization (CSTBO)

Despite having several advantages for solving optimization problems, the Sewing Training-Based Optimization Algorithm occasionally runs into problems. Every algorithm encounters a situation like this on occasion. In some challenging problems, this algorithm has the benefit of being able to escape the local minimum. Additionally, it can occasionally have a weak and raw convergence speed. Different approaches are used to solve this problem. Utilizing the benefits of another algorithm in addition to the current work is a useful method for this purpose. To produce even better results, the strengths of the Sewing Training-Based Optimization Algorithm and the particle swarm optimization (PSO) algorithm are combined in this study. Following the PSO algorithm [28], each individual working on a solution makes use of their knowledge as well as that of the other individuals to move up in the next movement. Two terms of position and velocity are crucial in this situation, according to the PSO algorithm. The mathematical definition of velocity is demonstrated by the following equation (Eqs. (12), (13), (14), (15), (16)):

(12) $$v_{new}=c_{1}\left(Z_{i}^{localbest}-Z_{i}\right)+c_{2}\left(Z_{i}^{globalbest}-Z_{i}\right)+wv$$

where, $c_{1}$ and $c_{2}$ are the moving factors for the candidates for the local and global best with a solution and the previous particle velocity, v and $v_{new}$ are the preceding and the present, in turn, particle velocities, and $Z_{i}^{localbest}$ and $Z_{i}^{globalbest}$ represent the descriptions of the current best position and the global best position for optimization. Then, by combining the PSO updating equation with the use of a weighting formula, the new position can be updated as follows [29]:

(13) $$Z_{i,j}^{*}=Z_{i,j}+\alpha \times ({lb}_{j}+r_{i,j}\left({ub}_{j}-{lb}_{j}\right)/t+\beta \times v_{new}$$

Accordingly, the final updating equation can be rewritten by the following equation:

(14) $$Z_{i,j}^{*}=Z_{i,j}+\alpha \times ({lb}_{j}+r_{i,j}\left({ub}_{j}-{lb}_{j}\right)/t+\beta \times \left[c_{1}\left(Z_{i}^{localbest}-Z_{i}\right)+c_{2}\left(Z_{i}^{globalbest}-Z_{i}\right)+wv\right]$$

where, this study considers α=0.45 and β=0.55 to provide more weight to the PSO-based exploration.

RETRACTED

### 2.3 DSTBO algorithm authentication

The proposed Combined *sewing training-based optimization* algorithm should be fairly analyzed to determine the effectiveness of the methods by applying them to some common benchmark functions and comparing the results with those obtained using other state-of-the-art methods [30]. In this case, we utilized six benchmark functions, including Unimodal, Multi-modal, and Hybrid which are listed in Table 1.

**Table 1:** Used benchmark functions in this investigation.

Type	Name	Test Function	Dim	Limitation	$F_{\min}$
Unimodal	Sphere	$F_{1}\left(x\right)=\sum_{i=1}^{n}x_{i}^{2}$	30	[-100,100]	0
	Schwefel2.22	$F_{2}\left(x\right)=\sum_{i=1}^{n}{|X}_{i}|+\prod_{i=1}^{n}\left|x_{i}\right|$	30	[-10,10]	0
Multimodal Basic Functions	Rosen brock’s	$F_{3}\left(x\right)=\sum_{i=1}^{n-1}\left[100{\left(x_{i+1}-x_{i}^{2}\right)}^{2}+{\left(x_{i}-1\right)}^{2}\right]$	30	[-30,30]	0
	Quartic	$F_{4}\left(x\right)=\sum_{i=1}^{n}{ix}_{i}^{4}+random[0,1)$	30	[-128,128]	0
Hybrid Benchmark Functions	Schwefe	$F_{5}\left(x\right)=\sum_{i=1}^{n}{-x}_{i}\;\sin\left(\sqrt{\left|x_{i}\right|}\right)$	30	[-500,500]	−418.9829
	Ackley	$F_{6}\left(x\right)=-20\;\exp\left(-0.2\sqrt{\frac{1}{n}\sum_{i=1}^{n}x_{i}^{2}}\right)\;–\;\exp\;\left(\frac{1}{n}\sum_{i=1}^{n}\cos(2\pi x_{i}\right))+20+e$	30	[-32,32]	0
	Schwefels Problem	$F_{7}\left(x\right)=\frac{\pi }{n}\left\{10\;\sin\left({\pi y}_{1}\right)+\sum_{i=1}^{n=1}{\left(y_{i}-1\right)}^{2}\left[1+10\;\sin^{2}\left(\pi y_{i+1}\right)\right]+{\left(y_{n}-1\right)}^{2}\right\}+\sum_{i=1}^{n}u\left(x_{i},10,100,4\right)$ $y_{i}=1+\frac{x_{i}+1}{4},u\left(x_{i},a,k,m\right)=\left\{ \begin{array}{cc} {k\left(x_{i}-a\right)}^{m} & x_{i}>a\\ 0 & -a<x_{i}<a\\ {k\left(-x_{i}-a\right)}^{m} & x_{i}<-a \end{array}\right.$	30	[-50,50]	0

To demonstrate the method’s effectiveness, it should be compared to some cutting-edge techniques. In this case, three metaheuristic algorithms, including Wildebeest herd optimization (WHO) [31], Archimedes Optimization Algorithm (AOA) [32], World Cup Optimization (WCO) [33], and the original Sewing Training-Based Optimization are compared for further clarification. Table 2 lists the parameters that were set for the algorithms in this study. It should be noted that determining the best value for the variables of a metaheuristic is an important and challenging task. A more systematic approach is to use techniques such as grid search, random search, or Bayesian optimization to explore the space of possible parameter values and identify those that lead to the best performance. These methods can help to reduce the amount of manual effort required and improve the efficiency of the parameter tuning process. However, it’s important to keep in mind that even with these techniques, parameter tuning can still be a complex and iterative process that requires careful consideration and evaluation of the results. Ultimately, the choice of parameter values will depend on the specific problem being solved and the characteristics of the metaheuristic being used. A simpler method that is performed in this study is to use the Trial and error method. This method can be a useful strategy for finding good values, but it can also be time-consuming and may not lead to the best results. However, the parameter of the other comparative methods is considered as much as possible by default for better observations.

RETRACTED

**Table 2:** Set parameters for the algorithms in this study.

Algorithm	Parameter	Value
WHO [31]	$\alpha_{1}$	0.9
	$\beta_{1}$	0.3
	$\alpha_{2}$	0.2
	$\beta_{2}$	0.8
AOA [32]	Protection probability	10%
	Elimination probability	25%
	$c_{1}$	1.5
	$c_{2}$	1.5
WCO [33]	Playoff	0.04
	ac	0.3

Table 3 shows the results of the simulation and a comparison of the suggested combined sewing training-based optimization based on average value (AVE) and standard deviation value. It should be noted that the method will have better accuracy and convergence speed through the analysis if the study’s AVE and STD values have lower results [34]. The comparison between the proposed Combined Sewing Training-Based Optimization and the other methods under study is shown in Table 4.

**Table 3:** Comparison of the proposed Combined Sewing Training-Based Optimization algorithm with the other methods under consideration.

Function	Algorithms					
	WHO [31]		WHO [31]		AOA [32]	
	**Mean**	**STD**	**Mean**	**STD**	**Mean**	**STD**
$F_{1}$	6.23 E−8	10.92E−8	5.52 E−9	9.38–9	4.95 E−10	6.83E-10
$F_{2}$	10.59E−5	12.83E−5	15.41E−6	18.81E−6	13.55 E−7	15.93E-7
$F_{3}$	1.83	1.59	1.78	1.33	1.16	1.096
$F_{4}$	8.14E−5	3.025E−5	5.003E−6	8.025E−6	6.083E-7	8.015E-7
$F_{5}$	−275.38	58.59	−315.34	48.8	−3982.64	43.01
$F_{6}$	9.98E−9	14.93–9	23.83E-9	32.58E-9	10.88E-10	8.92E-10

Function	Algorithms			
	**STBO** [27]		**CSTBO**	
	**Mean**	**STD**	**Mean**	**STD**
$F_{1}$	5.69 E−11	8.49E−11	6.91 E−12	9.27E-12
$F_{2}$	12.71 E−7	14.74E−7	11.38E−8	12.39E-8
$F_{3}$	1.059	0.91	0.83	0.12
$F_{4}$	18.082E−7	20.009E−7	3.048E−8	7.011E-8
$F_{5}$	−352.89	40.23	−386.81	26.12
$F_{6}$	11.06 E−11	19.005E−11	8.49 E−12	12.28E-12

**Table 4:** Error-values of the contrasting tactics.

#	Method	Type	MSE
1	LSTM network [35]	Forecasting of the Short-term electricity	0.71
2		Forecasting of the Medium-term electricity	0.62
3		Forecasting of the Long-term electricity	0.65
4	ENN/GA [26]	Forecasting of the Short-term electricity	0.53
5		Forecasting of the Medium-term electricity	0.55
6		Forecasting of the Long-term electricity	0.58
07	FNGB [36]	Forecasting of the Short-term electricity	0.60
8		Forecasting of the Medium-term electricity	0.61
9		Forecasting of the Long-term electricity	0.55
10	SqueezeNet/CSTBO	Forecasting of the Short-term electricity	0.48
11		Forecasting of the Medium-term electricity	0.49
12		Forecasting of the Long-term electricity	0.53

Table 3’s findings show that the proposed Combined Sewing Training-Based Optimization algorithm provides the highest accuracy. These results show that the proposed method outperforms the alternatives in terms of solving the benchmark functions under study. By examining the standard deviation value of these methods, we can further see that the suggested approach produced one of the minimal results. This demonstrates the opposition procedure’s higher reliability throughout various runs in comparison to other examined techniques and its improved dependability in addressing optimization issues. As a result, the proposed Combined Sewing Training-Based Optimization algorithm can be used as a useful tool for CNN placement that will produce a trustworthy forecasting tool.

RETRACTED

## 3 Optimized SqueezeNet structure by CSTBO algorithm

### 3.1 SqueezeNet structure

Due to their high effectiveness, convolutional neural networks (CNNs), as a popular deep learning technique, are now widely used in a variety of applications. For the artificial processing and forward classification of multidimensional data, such as images, convolutional neural networks were developed [37]. To better mimic the operation of the human visual system, its structure has been updated.

Similar to other artificial neural networks, convolutional neural networks are composed of neurons that store biases and weights and contain a decision-making process in the following layers [38]. The hidden layers' size will be very large, and its updating process will take a very long time if fully connected layers and normal neural networks for image classification have been used.

Convolutional neural networks have a lot of parameters, which rises memory usage. SqueezeNet is an architecture that is identical to the AlexNet architecture but has fifty times fewer parameters, making it ideal for gadgets like mobile phones. An activation, convolution, and pooling function are all combined to form a convolution layer.

Global average pooling is a technique used in the SqueezeNet in place of their customary fully connected layer. In contrast to networks that add a fully connected layer for classification, this method creates a feature map for each class after the final mlpconv layer rather than adding a full layer as is done in networks that use the fully connected layer. They are interconnected on top of feature maps, gaining from them, and the results of feature vector analysis are fed directly into Softmax. Due to the lack of optimization parameters, one advantage of this layer is that it does not cause more trouble than it solves. Alternatively, the Softmax is extra resilient to local variations and more in line with the concept of convolution networks.

RETRACTED

The SqueezeNet is composed of various fire modules, each of which has a squeeze convolution layer and an expansion layer. The SqueezeNet Fire Module is illustrated in Fig. 1.

**Fig. 1:** Fire module of a SqueezeNet.

The squeeze convolution layer’s findings are passed on to the following expand layer in the fire modules, as seen in Fig. 1. The SqueezeNet also starts with a single convolution layer, goes across eight Fire modules, and finishes with a final convolution layer. Moreover, SqueezeNet performs the max pooling operation in two steps, as shown in Fig. 2.

**Fig. 2:** Structure of a SqueezeNet.

### 3.2 Optimized SqueezeNet based on CSTBO algorithm

As mentioned before, when training SqueezeNet, the CSTBO algorithm is employed. This method can offer and improve the potential resolution to the specified optimization problems. The phases of the *CSTBO algorithm* are outlined below.

It is necessary to initialize the algorithmic restrictions and solutions before using them to generate the optimum solution. The stated aim function is to identify the MSE’s ideal solution, such that [39]:

(15) $$Fit=\frac{1}{M}\sum_{j=1}^{M}{\left(D_{j}-Y_{j}\right)}^{2}$$

where, M determines the total sample quantity, and $D_{j}$ and $Y_{j}$ signify the desired value and the output of the SqueezeNet.

The goal of this idea is to minimize the fitness function using the CSTBO algorithm, in other words:

(16) minFit

## 4 Dataset description

The data used in the simulation was taken from the 2022 report “Uk Energy In Brief 2022” [40]. Confirmation, training, and test sub-data were taken from the input data to provide a proper analysis. The acquired dataset is sufficient to carry out the suggested optimized SqueezeNet forecasting because it includes the required scheduling types, such as Short, Long, and Medium-Term Forecasting.

Because it better satisfies the SqueezeNet model, a day-in-advance prediction with a 30-min precision is employed. Input, goal parameters, and invisible layer neurons are assigned before the experiment. Input variables include day, month, and year. By identifying and employing a hidden layer, the experiment aims to improve the accuracy and correctness of network training. The variable about power usage serves as a goal variable for the duration of the experiment.

RETRACTED

The findings are divided into three categories of daily energy consumption pattern, consumer short-term, and long-term forecasting.

### 4.1 Summertime energy consumption

Fig. 3 displays a weekday energy consumption curve for the summer. An hourly representation of this pattern is shown.

It is evident from Fig. 3 as well as Fig. 4, due to the heavy use of cooling equipment (that is, air conditioner). Fig. 4 depicts a pattern of holiday energy consumption. Another way to describe this pattern is on an hourly basis.

**Fig. 3:** Weekday energy consumption curve for summer.

**Fig. 4:** Pattern of holiday energy consumption.

Summer vacations show a trend in energy consumption that is a little lower than working days. The prolonged sunny day also contributes to the negligibly good results that green power systems produce.

### 4.2 Using electricity in the winter

Fig. 5 displays the winter’s energy usage during the workweek. An hourly representation of this pattern is shown.

**Fig. 5:** Winter energy usage patterns on weekdays.

Fig. 6 depicts the winter holiday power consumption curve. On an hourly basis, this pattern can also be described.

**Fig. 6:** Winter holiday power consumption curve.

Findings of Fig. 5, Fig. 6 demonstrate that, particularly at night when heating devices are used, wintertime power usage is marginally higher than summertime usage. Additionally, it is asserted that the power generated by renewable energy sources is less than on a summer day because of the typical sunny or cloudy day. Furthermore, it can be inferred from Fig. 3, Fig. 4, Fig. 5, Fig. 6, the patterns of energy consumption and the production of renewable energy sources during the summer are slightly different from those during the winter.

## 5 Simulation results

### 5.1 System formation

Experiments are performed by Matlab R2018b on a laptop with a core i7-6700HQ Asus N552 processor and 12 GB RAM. It is assumed that there will be a maximum of 200 iterations and that there will be 60 individuals. Energy forecast performance is enhanced by using the suggested SqueezeNet method. To meet consumer energy demand and to better understand how customers use energy, the predicted electricity under the proposed SqueezeNet method is used. The offered optimized SqueezeNet/CSTBO method is compared to some other techniques in the literature, such as the LSTM network [35], Elman neural networks with evolutive optimization (ENN/GA) [26], and fractional nonlinear grey Bernoulli model (FNGB) [36].

### 5.2 Forecasting of the daily energy demand

Fig. 6 shows a projected daily energy use for a typical day and illustrates the consumer power usage patterns over time. A time window has been set up to collect the objective and input data from the customer at intervals of 20 min, allowing for highly effective neural network training. The results of comparing predicted and actual energy demand are shown in Fig. 7.

RETRACTED

**Fig. 7:** Energy projection for a typical day.

The study has made predictions about energy demand and compared them with the actual energy demand. Assuming that the authors' results provide the best results means that the authors have used the most accurate and reliable methods for predicting energy demand and have obtained the most accurate and reliable data for actual energy demand. Therefore, the results presented in Fig. 6 are considered to be the most valid and trustworthy representation of the comparison between predicted and actual energy demand. However, it is important to note that scientific research is subject to ongoing debate and review, and the validity of any particular study’s results may be challenged or revised as new data and methods become available. It is always a good practice to critically evaluate the methodology and data sources used in any scientific study and consider the limitations and uncertainties associated with the findings.

### 5.3 Forecasting of the monthly energy demand

The expected and actual monthly kilowatt usage for energy is shown in Fig. 8. The graphs display the trends in demand and consumption for the suggested SqueezeNet/CSTBO, ENN/GA [26], and FNGB [36].

**Fig. 8:** Typical day’s projected energy consumption for the month.

The statement is describing the results obtained from an experiment or study related to energy consumption forecasting using the SqueezeNet/CSTBO technique. The results are referring to Fig. 7, which presumably presents the results of the study, to support the claim that the suggested technique has a low error rate when compared to other comparable algorithms. Moreover, the statement indicates that the suggested technique, i.e., SqueezeNet/CSTBO, has demonstrated a high degree of accuracy in forecasting short-term energy consumption. This suggests that the technique can be useful for predicting future energy consumption patterns, which can help organizations or individuals make informed decisions regarding energy usage, resource allocation, and cost-saving measures.

### 5.4 Forecasting of the annual energy demand

The projected and actual yearly kilowatt usage is shown in Fig. 9. The graphs display the trends in demand and consumption for the suggested SqueezeNet/CSTBO, ENN/GA, and FNGB.

**Fig. 9:** A projection of the annual energy use for a typical day.

RETRACTED

### 5.5 Comparing the outcomes of optimization

For both short- and long-term power forecasting, the suggested optimization approach’s convergence values were compared to those of the other second-best method, i.e., FNGB. The results are shown in Fig. 10, Fig. 11. The cost value in the FNGB is not the best or most ideal solution for forecasting short-term energy.

**Fig. 10:** Values of optimization convergence for FNGB method versus short-term energy prediction.

**Fig. 11:** Long, medium, and short-term power forecasting optimization convergence values compared with the FNGB method.

The research mentioned above for the example under discussion demonstrates that using the proposed SqueezeNet/CSTBO method results in cost values for short-term energy prediction that are significantly lower than those obtained using the FNGB. So, it could be said that the suggested SqueezeNet/CSTBO and FNGB algorithms result in better convergence outcomes for both short-term power forecasting and long-term energy predicting.

As a result, the suggested SqueezeNet/CSTBO may be the main consideration for processes of medium-term power prediction and long-term energy prediction. As a result, the suggested SqueezeNet/CSTBO and FNGB algorithms for altering the NN method weight worked well and produced better results for demand forecasting.

According to the results, the SqueezeNet/CSTBO procedure has yielded the best results when compared to other prediction methods that have been evaluated, and the results are truly satisfying. The evaluation has been performed based on the Mean Squared Error (MSE) metric, which is a commonly used metric in regression problems. MSE measures the average squared difference between the predicted and actual values. The lower the value of MSE, the better the model’s performance. The results show that the SqueezeNet/CSTBO procedure has the lowest MSE across all prediction types. This implies that the model is performing well in predicting various types of data. The statement suggests that the results are truly satisfying, indicating that the model has performed exceptionally well.

## 6 Conclusions

Accurate forecasting of the consumption curve for network load management and dispatching has become crucial for distribution businesses with the emergence of smart networks. Distribution firms face significant difficulty in the development and selection of time series models to select the best and most useful model for load forecasting. The objective of this article was to develop an optimal load forecasting model utilizing machine learning on short, long, and medium loads an optimized version of SqueezeNet based on an improved metaheuristic, called a customized version of the Sewing Training-Based Optimizer (CSTBO) with the forecasting models' parameters for load forecasting based on distribution network information. Here, the proposed SqueezeNet/CSTBO method and those of some other published techniques were then implemented after the method to a case study with three different types of demands-short, long, and medium-term. The results demonstrated that employing the suggested technique was a viable option for energy consumption forecasting. In conclusion, the proposed method offers several advantages over existing techniques in electric load forecasting. Its high accuracy, ability to handle different types of demands, and real-time analysis make it a viable option for energy consumption forecasting. However, the potential for data bias and the need for real-time data should be taken into consideration when implementing the method in practice. The main results of this study are as follows:

− The proposed technique was demonstrated as a viable option for energy consumption forecasting
− The study showed that the proposed SqueezeNet/CSTBO method outperformed other published techniques for short-term load forecasting
− The proposed SqueezeNet/CSTBO method had a competitive performance for medium-term and long-term load forecasting compared to other published techniques.

RETRACTED

## Declaration of competing interest

The authors declare that they have no known competing financial interests or personal relationships that could have appeared to influence the work reported in this paper
